# A Six-Gene Risk Model Based on the Immune Score Reveals Prognosis in Intermediate-Risk Acute Myeloid Leukemia

**DOI:** 10.1155/2022/4010786

**Published:** 2022-04-29

**Authors:** Cong Lu, Dong Hu, Jin'e Zheng, Shiyi Cao, Jiang Zhu, Xiangjun Chen, Shiang Huang, Junxia Yao

**Affiliations:** ^1^Center for Stem Cell Research and Application, Union Hospital, Tongji Medical College, Huazhong University of Science and Technology, Wuhan 430022, China; ^2^Institute of Hematology, Union Hospital, Tongji Medical College, Huazhong University of Science and Technology, Wuhan 430022, China; ^3^School of Public Health, Tongji Medical College, Huazhong University of Science and Technology, Wuhan, 430030 Hubei, China

## Abstract

Tumor microenvironment (TME) has been revealed as an important determinant of diagnosis and treatment response in AML patients. The scores of immune and stromal cell scores of AML in the intermediate-risk group from The Cancer Genome Atlas (TCGA) database were calculated using the Estimation of STromal and Immune cells in MAlignant Tumor tissues using Expression data algorithm. Differentially expressed genes were identified between high and low scores. Gene set enrichment and pathway analyses were performed. A risk score model based on TME for six immune-related genes was established and validated. Patients with a lower immune score had a longer overall survival than those with a higher score (*P* = 0.044). A total of 805 intersected genes as differentially expressed genes were identified and selected according to the comparison of both immune and stromal scores. The functional enrichment analysis shows that these genes are mainly associated with the immune/inflammatory response. The risk score model based on TME for six immune-related genes (including MEF2C, ENPP2, FAM107A, CD37, TNFAIP8L2, and CASS4) was established and validated in the TCGA database and well validated in the TARGET database (*P* = 0.005). A key microenvironment-related gene signature was identified that affects the outcomes of AML patients in the intermediate-risk group and might serve as therapeutic targets.

## 1. Introduction

Acute myeloid leukemia (AML) is a highly heterogeneous and urgent hematopoietic malignancy. Genetic abnormalities in hematopoietic progenitors eventually lead to tumorigenesis in immature myeloid cells [1]. Patients are usually mainly stratified according to genomic risk factors based on their initial disease status [2, 3]. Treatment regimens especially in postremission consolidation therapy were significantly different among patients with different risk stratifications [4]. As patient-related and disease-related factors contribute to the individual's response to treatment and long-term survival, the disease prediction more accurately for AML patients is essential. Although individualized precision therapy has made some progress, it is still not enough to meet the needs of AML patients, especially for the patients in the intermediate-risk group. Therefore, new molecular biological indicators are still needed to refine and guide the treatment and prognosis of patients.

Tumor initiation is influenced by the host immune system, and immunological biomarkers are becoming more and more important for prognosis prediction. It has been proposed that the immune scoring staging system is applied to solid tumors to predict the prognosis of solid tumors [5–7]. Tumor microenvironment (TME) has been revealed as an important determinant of diagnosis and treatment response in cancer patients. The high complexity of TME is reflected in multiple interactions among tumor, stromal, immune, and mesenchymal cells through changes in some soluble factors and extracellular matrix components [8, 9]. Immune and stromal cells are considered to play a pivotal role in disease progression and prognosis assessment [10].

Yoshihara et al. designed an algorithm called Estimation of STromal and Immune cells in MAlignant Tumor tissues using Expression data (ESTIMATE) which is an algorithm used to estimate and sequence populations of immune and stromal cells within TME to assess nontumor cell invasion by analyzing specific gene expression characteristics [11]. This algorithm has been successfully applied to the analysis of immune-related characteristics of some solid tumors, such as breast cancer [12], prostate cancer [13], and colon cancer [14]. However, only a few reports have used the ESTIMATE algorithm in the analysis of AML patients to reveal the mechanism of bone marrow immune microenvironment and find some special immune-related genes in AML patients [15, 16].

In this study, we used this algorithm to analyze the bone marrow microenvironment of AML patients in the intermediate-risk group. We have found some immune-related genes and constructed a risk score prognosis model based on TME, which is aimed at finding new immune-biological molecular markers to guide the precise prognosis and treatment of patients in intermediate-risk AML.

## 2. Materials and Methods

### 2.1. Data Source

From The Cancer Genome Atlas (TCGA) database, we downloaded the RNA-Seq data of AML patients in the intermediate-risk group and corresponding clinical profiles. 81 AML patients of the intermediate-risk group were included in this analysis. Using the ESTIMATE algorithm, we obtained the immune scores of the AML patients screened and the stromal scores of chosen samples were calculated [11]. Meanwhile, 129 AML patients in intermediate-risk group from the TARGET database were extracted for external validation.

### 2.2. The Identification and Obtaining of Differential Gene Expression (DEGs)

ESTIMATE is defined as the use of the unique properties of the cancer sample transcription profile to infer the contents of tumor cells as well as the different infiltrating normal cells [11]. We installed the ESTIMATE package using R software by reading transcriptome files.

The scores based on TME for each AML sample were calculated. All the enrolled AML patients chosen were identified as high-/low-score groups according to the median scores. Data analysis was performed with the R package limma [17]. In this study, DEGs were selected based on adjusted *P* value < 0.05 and absolute fold change > 1. The heatmaps of the DEGs were drawn using R language.

### 2.3. Gene Enrichment and Pathway Analyses

Gene set enrichment and pathway analyses were performed using the R package clusterProfiler (Bioconductor package version 3.8) for the obtained differential genes [18].

### 2.4. Protein Network Construction

As a powerful tool for analyzing protein network interactions, STRING (http://www.string-db.org/) was exploited to explore potential relationships among DEGs [19]. We reconstructed the network using Cytoscape software [20].

We imported the PPI Web figure of 361 DEGs generated by STRING into Cytoscape software. The cytoHubba plugin in Cytoscape software was used for hunting the top 30 nodes of genes known as hub genes. The number of nodes for each hub gene can be calculated by the software or by R. We ranked hub genes by the degree from low to high.

### 2.5. Risk Scoring Model Construction

First, the survival-related DEGs were screened and identified by the log-rank test using the survival R package from all the genes using the following two models [21]. Then, we used univariate cox regression analysis and Lasso regression to screen survival-related genes included in the model from the genes chosen in the first step [22]. Lasso regression was used to avoid overfitting. The candidate mRNAs were subjected to multiple proportional risk regression to construct a risk scoring model: risk score (patient) = ∑*I* coefficient (mRNAi)∗expression (mRNAi).

### 2.6. Nomogram Drawing

We drew a nomogram to predict the survival rate of the constructed model. The immune genes screened from the risk score model were used to construct. A patient's score was first derived from the coefficients of individual immune genes in the model. The corresponding score for each immune gene is then added up to get a total score. Patient's survival was predicted according to the length of the line corresponding to the total score.

All analyses were performed by R 4.0.2 and Bioconductor package version3.8.

## 3. Results

### 3.1. Association of Immune and Stromal Scores with Clinical Characteristics of AML Patients in the Intermediate Risk Group

81 AML patients in the intermediate-risk group were retrieved from the TCGA database. Their clinical characteristics and immune/stromal scores were shown in Table 1. There were 38 female cases (46.3%) and 44 male cases (53.7%). According to classification of the FAB subtype, there were 6 cases of M0 (undifferentiated subtype), 21 cases of M1, 23 cases of M2, 18 cases of M4, and 11 cases of M5. Each of the other subtypes has only one case. The scores of these patients calculated using ESTIMATE displayed that the value of immune scores ranged from 1577.53 to 3094.61, while stromal scores ranged from −1644.36 to 4140.67. The median values of patients for clinical characteristic were listed in Table 1. We, respectively, made an analysis about the age, gender, FAB subtype, and *FLT3*/*NPM1* gene mutations in relation to immune scores between the two groups. The results showed that the immune score was higher in older patients (*P* = 0.041) but not correlated with the FAB subtype or gene mutations (*P* > 0.05).

### 3.2. Differential Expression Gene Screening Based on the Immune Score

To assess the correlations between the scores and overall survival (OS) in intermediate-risk AML patients, the patients were then separated into the high- or low-score group. We found that the OS in patients with a lower immune score were longer than those in patients with a higher immune score (*P* = 0.044, Figure 1(a)). At the same time, patients with a low stromal score had longer OS than those with a high stromal score but the difference was not significant (*P* = 0.615, Figure 1(a)).

In order to find the differential expression genes in the immune microenvironment, 81 AML patients were divided into two groups based on the median immune score. The high- and low-score groups showed different gene expression patterns (Figure 1(b)), suggesting that gene expression profiles may be used to describe differences between the two groups. According to the comparison of immune scores, 1173 genes were upregulated and 406 genes were downregulated. At the same time, 1020 genes were upregulated and 442 genes were downregulated between the high- and low-stromal score groups (|log *FC*| > 1, FDR < 0.05). Furthermore, common differentially expressed genes in the high-expression group and the low-expression group were analyzed. A total of 710 genes were upregulated and 95 genes were downregulated (Figure 1(c)). We selected these 805 intersected genes as DEGs for subsequent analysis to explore their correlation with the BM microenvironment in intermediate risk of AML.

### 3.3. Functional Pathway Enrichment Analysis

To investigate the identified genes' functions, we used the R language clusterProfiler package to conduct the GO term and KEGG path enrichment analysis (corrected *P* value < 0.05). There were 698 GO items of the biological process (BP), 64 GO items of the molecular function (MF), and 46 GO items of the cellular component (CC).

In terms of the first 30 GO biological processes, DEGs are mainly concentrated in regulating the immune response process, cytokine secretion, inflammatory response, and tumor necrosis. The biological processes of these DEGs mainly include T cell activation, leukocyte proliferation, lymphocyte activation regulation, leukocyte adhesion between leukocytes, and leukocyte migration and regulation (Figure 2(a)). Molecular functions include immunoglobulin binding, cytokine receptor activation, and mucopolysaccharide binding (Figure 2(b)).

In KEGG analysis, a total of 36 pathways were enriched, including hematopoietic generation associated with the blood system, tumor and immune processes, and correlation between cytokine receptors, such as the B cell receptor signaling pathway, Toll-like receptor, NF-*κ*B cell pathway, and HSA05221 myeloid leukemia directly associated with AML (Figure 2(b)).

### 3.4. Protein Network Interaction Analysis

To analyze the potential connection patterns between transcripts of the DEG gene set, the network between PPI (protein-protein interactions) was constructed by the STRING database. We loaded the PPI network from STRING with Cytoscape and a plugin called cytoHubba for flexible reconstruction (Figure 3(a)). The top 32 hub genes were listed as FPR2, C3, PTAFR, GNGT2, ITGAM, CKAP4, FPR1, HLA-DQA1, HLA-DQB1, HLA-DRB5, CXCL10, CYBB, FCER1G, FCGR1A, PSAP, CCR1, CCR2, CCR5, CLEC4D, FCAR, C5AR1, CCL1, CX3CR1, CXCL16, IL10, IRF4, LILRB2, P2RY13, S1PR3, LYZ, PTPRJ, and TNFRSF1B (Figure 3(b)). It should be noted that most of these key nodes are composed of proteins/genes involved in immune regulation. The subnetwork was composed by 32 hub genes screened. The rank of the edges according to degree was shown in Figure 3(c).

### 3.5. Establishment of a Risk Score Model for Immune-Related Prognostic Genes

To establish a risk score model for prognostic genes, 92 differentially expressed genes were first filtered and screened using univariate Cox analysis. There were 63 survival-related key DEGs that showed statistically significances in the univariate analysis (*P* < 0.05). According to the Lasso regression and multivariate Cox regression analysis, 6 independent predictors entered the risk scoring model. The coefficient and crossvalidation of Lasso regression were shown in Figure 4(a). There were 6 genes that entered into the multifactor risk regression model: MEF2C, ENPP2, FAM107A, CD37, TNFAIP8L2, and CASS4. The forest map of the multivariate Cox regression model was shown in Figure 4(b). The concordance index was 0.78.

The risk scoring model was constructed as follows: riskscore = 1.064015∗(MEF2C)exp + 1.215766∗(ENPP2)exp + 9.98*E* − 05∗(FAM107A)exp + 1.020001∗(CD37)exp + 1.027994∗(TNFAIP8L2)exp + 1.192386∗(CASS4)exp.

After we obtained the immune-related gene risk score model, we calculated the risk value of each AML patient in the intermediate-risk group based on the expression of the model candidate gene for each patient. According to the median value, patients were divided into two groups. There were significant differences in survival curves between the two risk groups (*P* < 0.001). The areas under the ROC curve of 1-/2-/3-year survival rates were 0.893, 0.907, and 0.882, respectively (Figure 4(c)). We plotted the nomogram of the constructed gene risk model. The score of each risk gene can be obtained through the array diagram, and a corresponding score can be obtained according to the expression level of each risk gene. Then, the scores can be added together to obtain a comprehensive score, and then, the final score can be corresponding to the survival line to obtain the 1-year, 2-year, and 3-year survival rates of the patient (Figure 4(d)).

### 3.6. Risk Score Model Validated in TARGET

Gene expression and survival information of 129 AML patients in intermediate cytogenetic risk from the TARGET database were extracted. The risk score for each sample in TARGET was calculated based on the immune gene risk score formula established. The results showed that there were significant survival differences between the two groups (*P* = 0.005, Figure 5). It suggested that the immune-gene risk score model was well validated in the TARGET database.

## 4. Discussion

AML is one of the most common hematopoietic malignancies in adults [23]. The therapeutic options and prognosis of patients is highly varied among AML patients [24]. Especially among patients in the intermediate cytogenetic risk group, the choice of treatment and prognosis are heterogeneous and even difficult to choose. Bone marrow TME plays a crucial role in the development, progression, and clinical outcome of AML. In this study, we used the ESTIMATE algorithm to identify TME genes and construct an immune-related risk score model which could predict the clinical outcome in patients with AML in the intermediate-risk group from the database of TCGA.

As pointed out, immune scores were associated with survival and prognosis in patients with AML or solid tumor. It may be due to the different signaling pathways triggered by these immune-related gene groups, which is worthy of further discussion and research.

According to the median score value, we made an analysis of correlation between parts of clinical features and immune scores. As a result, we found that the immune score was only associated with age, but neither with *FLT*3 or *NPM*1 gene mutation nor with the FAB subtype. We speculated that the correlation between the immune score and known prognostic gene mutations remains unclear in patients with AML in the intermediate-risk group, which is worth further study by expanding the sample size.

The relationship between the survival time and immune/stromal score was calculated separately. The results showed that the survival time in the low-score group was significantly longer than that in the high-score group. Huang et al. found that the OS in the high-score group was shorter [15]. Ni et al. revealed that a higher immune score and ESTIMATE score were associated with worse OS days [25]. These observations were consistent with our research, which suggested that patients with high immune scores have worse prognostic outcomes. We inferred that the immune score might be an adverse prognostic factor in AML. Studies have also shown a correlation between immune scores in the tumor microenvironment and survival in solid tumors [26].

In order to find out the reasons for the differences in survival and clinical characteristics between the two score groups, we conducted functional enrichment analysis of the DEGs in the intersection of the two parts. The results showed that the DEGs were mainly concentrated in T cell activation and proliferation, globulin secretion, and cytokine receptor interaction. They also participated in cytokine-cytokine receptor interaction, chemokine signaling pathway, Toll-like receptor signaling pathway, NF-*κ*B signaling pathway, and AML-related pathway HSA05221. These analyses indicate that these differential genes may participate in a critical part in AML initiation and merit further verification of the function of related differential genes by molecular experiment. These may provide some research ideas in the pathogenesis of AML on immunology.

A total of 96 DEG genes were associated with OS in patients with AML in the intermediate-risk group. After multiple regression analysis, we finally established a six-TME-related gene model. It was validated in a separate cohort of target-AML patients. In the gene risk score model based on TME, a total of six candidate genes were identified, including MEF2C, ENPP2, FAM107A, CD37, TNFAIP8L2, and CASS4. Not only was a single gene of the risk-score model associated with survival in patients with AML in intermediate risk separately, the model also could be used to predict the outcome of AML patients in the intermediate-risk group.

MEF2C is one member of the MADS transcription factor family. It is involved in the regulation of self-renewal and differentiation for the hematopoietic system [27]. Recent studies have focused on improving targeted therapies in AML [28]. Brown et al. [29] used high-precision mass spectrometry to indicate that high levels of phosphorylated MEF2C S222 are obviously associated with chemotherapeutic resistance observed in a cytogenetic normal and MLL-recombinant leukemia cohort. This verifies that MEF2C phosphorylation may promote chemotherapy resistance and its blocking could be used to improve AML treatment. Tarumoto et al. [30] used a CRISPR screening to reveal the important role of LKB1 and its salt-induced kinase effector (SIK3 and SIK2 partial redundancy) in maintaining MEF2C function in AML. It was found that MEF2C-dependent leukemia was sensitive to chemical inhibition-targeted SIK activity.

ENPP2 (ectonucleotide pyrophosphate phosphodiesterase 2) is an enzyme present in blood circulation that functions both as a phosphodiesterase and as a phospholipase. This gene product stimulates the motility of tumor cells, which is upregulated in several kinds of carcinomas [31]. In an analysis of 672 normal karyotype AML patients, an analysis between FLT3-ITD and FLT3-TKD revealed a distinct difference for STAT5 target gene expression as well as deregulation of ENPP2 [32].

CD37 is a transmembrane protein of the 4 superfamily that plays a role in the regulation of cell activation, growth, and motility in mediating signal transduction events [33]. It has been focused as a therapeutic target recently. In the analysis of CD37 expression in normal tissues and malignancies, it was found to be expressed in T cell lymphoma and AML [34]. They developed an antigen drug called AGS67E-binding compound targeting CD37 for the treatment of B/T cell malignancies. It demonstrated that CD37 was well expressed in AML and is a potential drug target. The results of Zhang et al.'s research showed that mRNA expression of CD37 was significantly upregulated in patients with AML compared with healthy controls [35]. The result showed that patients with high CD37 expression had shorter OS and disease-free survival (DFS), which was in some agreement with our conclusion.

By identifying differential genes, we established and validated a risk score model based on TME for six immune-related genes. In these genes, MEF2C and CD37 could be novel immune tumor markers associated with prolonged survival in AML and may have an important relationship with the tumorigenesis and progression of AML. We hope that our findings will contribute to better guidance of prognosis and treatment for AML in the intermediate-risk group.

## Figures and Tables

**Figure 1:** The differentially expressed genes (DEGs) of the immune score and stromal score. (a) The survival analysis between low- and high-score groups. (b) Heat maps between high- and low-score groups. (c) Common DEGs of upregulated and downregulated DEGs.

**Figure 2:** The functional enrichment analysis of DEGs. (a) GO dotplot. (b) KEGG dotplot.

**Figure 3:** Protein network interaction analysis of DEGs. (a) PPI by STRING. (b) 33 hub genes screened by cytoHubba. (c) The rank of the edges.

**Figure 4:** The construction and analysis of the risk score model. (a) The coefficients and partial likelihood deviance of the Lasso regression. (b) The forest map of multivariate Cox. (c) The survival by Kaplan-Meier and ROC curves (1/2/3 years). (d) The nomogram of the constructed gene risk model.

**Figure 5:** The survival curve validated by TARGET database using Kaplan-Meier.

**Table 1:** The clinical characteristics and the immune score/stromal score.

Characteristic	Category	Cases	Immune score (median)	Stromal score (median)
Age	<60 years	45	2926.378	−914.957
	≥60 years	36	3233.629	−826.588

Gender	Male	43	3031.757	−881.792
	Female	38	3106.435	−925.398

FAB subtype	M0	6	3009.567	−833.614
	M1	21	2880.161	−1033.32
	M2	23	2901.244	−976.13
	M4	18	3243.899	−700.734
	M5	11	3274.568	−677.531
	M6	1	3511.771	−637.973
	M7	1	2684.707	−177.338

Karyotype	Normal	68	3070.489	−884.783
	Others	3	2998.283	466.029
	NA	10	—	—

FLT3 gene	Mutant	25	2930.084	−954.845
	WT	46	3096.285	−839.960
	NA	10	—	—

NPM1 gene	Mutant	28	3088.594	−918.332
	WT	43	3066.435	−872.269
	NA	10	—	—

## Data Availability

Publicly available datasets were analyzed in this study. This data can be found in the following: The Cancer Genome Atlas (https://portal.gdc.cancer.gov/).
